The article "Trends in Morphological Characteristics among 7- and 11-Year-Old Serbian Children: A Comparison between 1990 and 2020" was published in 2022. Journal: Biomed Res Int.

# Trends in Morphological Characteristics among 7- and 11-Year-Old Serbian Children: A Comparison between 1990 and 2020

**DOI:** 10.1155/2022/4070658

**Published:** 2022-09-29

**Authors:** Goran Đukić, Zlatko Ahmetović, Romana Romanov, Dušan Stupar, Goran Sporiš, Nebojša Trajković

**Affiliations:** ^1^Faculty of Sport and Psychology-Tims, Educons University, Novi Sad 21000, Serbia; ^2^Faculty of Kinesiology, University of Zagreb, Croatia; ^3^Faculty of Sport and Physical Education, University of Niš, Serbia

## Abstract

Since knowledge possession about the morphological characteristics trend is important to understand, it is necessary to monitor the physical growth and children's development. We have aimed to examine the current state, dynamics, and direction of changes in morphological characteristics, over a 30-year period in Serbian children and adolescents. Morphological characteristics measured in 2020 (*n* = 304; age 7 ± 6 and 11 ± 6) were compared with the results of same-age children and adolescents from 1990 (*n* = 1789). The following characteristics were measured: body height, body mass, body mass index, forearm circumference, and upper arm skinfold. The average height (95% IP) of 7-year-old boys was significantly lower in all morphological variables in 1990, compared to their 2020 peers, while in forearm circumference was opposite. As for the 11-year-old boys, body mass (*p* = 0.02) and BMI (*p* = 0.009) had significantly better average values in 2020 than 1990, whereas forearm circumference (1.6-2.5 cm) and upper arm skinfold (2.7-4.9 cm) results were opposite. Seven-year-old girls from a 1990 sample also had significantly lower average values for morphological characteristics, compared to their 2020 peers. All morphological characteristic variables of 11-year-old girls have significantly better average values in 1990 sample than in 2020, except for body mass (*p* = 0.47) and BMI (*p* = 0.55). The current results have presented a true “picture” of the trends in morphological characteristics status among 7- and 11-year-old Serbian children by comparing them with the already obtained results 30 years ago.

## 1. Introduction

Insufficient physical activity has been identified as a global key risk factor for mortality [1]. Hypokinesia, as a reduction in the activity of the musculoskeletal system, increases susceptibility to many diseases, as well as general energy use [2], which further leads to increased concern for children's health, mainly because of their daily activities and habits. In addition, we are coming to a confusing situation where new technological innovations and discoveries are undoubtedly helping people to do different types of work faster and easier, but no attention is paid to energy consumption, which definitely decreases [3]. Furthermore, some authors [4, 5] believe that children usually spend most of their free time sedentary, in front of an electronic device (TV, phone, tablet, computer, etc.). Also, reduced activity is associated with many eating habits that can cause energy imbalance and obesity, both in children and adolescents [2]. Although Ostojić et al. [6] believe that it is not unhealthy to be obese as long as a person is in good physical shape, they set the important question “Does obesity cause more damage to the human body than physical inactivity?”. Childhood obesity is expected to have more serious consequences for public health, given that being overweight in childhood usually continues into adulthood. Very poor fitness test results are also a crucial risk factor of diseases (diabetes, cancer, high blood pressure, osteoporosis, depression, anxiety etc.). Most of today's chronic diseases can be avoided only if quality upbringing and knowledge are passed onto children in early childhood, so that later, it can be implied with positive effect on adolescence and adulthood [2]. Given the worrying increase in hypokinesia in childhood, fundamental efforts should be made, in order to prevent long-term consequences [7]. Most public health recommendations actually encourage children and adolescents to exercise for at least 60 minutes of moderate to vigorous physical activity each day [1], so it is necessary to set another serious question, and it concerns which is whether children and adolescents meet the predefined criteria or not.

The article "Trends in Morphological Characteristics among 7- and 11-Year-Old Serbian Children: A Comparison between 1990 and 2020" was published in 2022. Journal: Biomed Res Int.

From birth to adulthood, a person's physical ability as well as physical development is influenced by many factors, both internal and external. We learn about the stages of development by monitoring the physical development and individual growth. Also, measuring and monitoring the children and adolescents growth are measured with the help of anthropometry [8]. It is necessary to monitor the physical growth and development of children, especially in the younger school age, because their body is subject to many external influences whose effects are felt only in the later period, which are very difficult to repair in later life [9]. Physical growth and development are first defined by body height and mass, while the crucial importance is the fact that in certain stages of ontogenetic growth and development, the influence and interaction of genetic factors in children is not the same. We associate morphological characteristics with bio-psycho-social status. It represents a set of characteristics that make up the constitution, body composition, structure, or assembly as an organized and relatively constant totality of characteristics in relation to each other. Also, endogenous factors represent internal factors, such as genetic and hormonal factors, while exogenous factors represent external factors, such as diet and physical activity [10].

The article "Trends in Morphological Characteristics among 7- and 11-Year-Old Serbian Children: A Comparison between 1990 and 2020" was published in 2022. Journal: Biomed Res Int.

Several authors have concluded that children who develop in more affluent conditions tend to have longer legs [11–13] and longer arms [12, 13], in relation to total body height. However, the results of changes in height and mass vary among countries in all socioeconomic groups [14], and the same changes are similar for both boys and girls [1, 15]. The prevalence of obesity and body size values has increased in most developed countries [15, 16], but in recent years, according to some authors [17, 18], the same parameters are only maintained. The prevalence of obesity was dominant in Eastern European countries compared to the rest of the continent and the United States [15]. It is purposefully recommended precisely because of its positive impact on many health aspects, body composition, cardiorespiratory fitness, mental health, attitude towards life, and even general physical activity [19]. Thus, the number of obese children and children with overweight is constantly increasing [20], children are increasingly moving, and thus, there is a slower development of motor skills.

Knowledge possession about the trends of morphological characteristics of children and adolescents is important to understand, given that they are related to many health outcomes. Also, the results may indicate a possible suppression of the negative trend [21], and in relation to the fact of high prevalence of increasing morphological characteristics, we can say that the current situation can be worrying [22]. Hence, we have aimed to examine the current state, dynamics, and direction of changes of secular trends in morphological characteristics, on a sample of 7- and 11-year-old Serbian children and adolescents, based on the first measurement that has been conducted 30 years ago.

## 2. Materials and Methods

### 2.1. Sample of Participants

The total participant sample was defined by the first measurement (*n* = 1789), conducted by Ahmetović et al. [23] in 1990. In order to ensure result comparability in 2020, the sample (*n* = 304) with same age (7 ± 6 months and 11 ± 6 months) was taken into consideration. Furthermore, the participants were taken from primary schools from Valjevo and Mionica. The number of participants in both time points is presented in Table 1.

### 2.2. Measurements

In order to examine the physical development, morphological variables were used at the first measurement: body height, body mass, body mass index (BMI), forearm circumference, and upper arm skinfold.

The article "Trends in Morphological Characteristics among 7- and 11-Year-Old Serbian Children: A Comparison between 1990 and 2020" was published in 2022. Journal: Biomed Res Int.

All measurement were conducted by the trained measurers, i.e., physical education teachers, as well as with the International Biological Program (IBP) recommendations [24]. In order to measure the defined variables, the following equipment was used in the measurement procedure: anthropometer by Martin, medical decimal weight, measuring tape (1 m long), and caliper.

If the time determinant is observed, this research is longitudinal and follows the time of 30 years (1990-2020), with the first research being conducted by the Ahmetović et al. [23]. The research was conducted in the school gymnasiums of the elementary school “Milan Rakić” from Mionica, primary school in Valjevo, and the fitness center “Top Form” Valjevo.

### 2.3. Statistical Analysis

Data will be presented as arithmetic mean (AS with 95% confidence interval (95% IP)) and standard deviation (SD). A participant sample from 1990 and 30 years later in the variables of morphological characteristics was compared with independent *t*-test tested whether statistically significant average difference (95% IP, standardized difference error (SE)) between the arithmetic means of the groups. Welch's test for unequal variance between groups was used as well. Differences between the years of sampling of morphological characteristics were assessed by individual *t*-test in children in relation to age and sex (7-year-old boys and girls, as well as 11-year-old boys and girls).

The level of inference was previously set at the level of *p* ≤ 0.05. Statistical analysis and graphical display were done using GraphPad [25] and Microsoft Excel [26].

## 3. Results

### 3.1. Morphological Characteristics of 7- and 11-Year-Old Boys (1990-2020)

In the 1990 sample, 7-year-old boys' height (95% IP) was between 127.2 and 128.3 cm, and body mass was from 26.82 to 27.74 kg, with BMI value of 16.91 ± 3.63 kg/m^2^. Their forearm circumference was between 17.58 and 17.88 cm, along with upper arm skinfold from 8.2 to 8.9 cm. Furthermore, 11-year-old boys' height (95% IP) was between 146.9 and 148.2 cm, and body mass was from 39.5 to 41.2 kg, with BMI value of 18.67 ± 4.11 kg/m^2^. Their forearm circumference was between 20.1 and 20.4 cm, along with upper arm skinfold from 10.3 to 11.3 cm. In the 2020 sample, 7-year-old boys' height (95% IP) was between 130.53 and 132.92 cm, while body mass ranged from 29.93 to 33.86 kg, with BMI value of 18.58 ± 3.57 kg/m^2^. Their forearm circumference was between 18.85 and 18.02 cm, along with upper arm skinfold from 13.78 to 16.00 cm. Furthermore, 11-year-old boys' height (95% IP) was between 146.2 and 149.2 cm, and body mass ranged from 41 to 45.2 kg, with BMI values 19.93 ± 4.71 kg/m^2^. Their forearm circumference was between 21.81 and 22.71 cm, along with upper arm skinfold from 13.63 to 15.52 cm.

The article "Trends in Morphological Characteristics among 7- and 11-Year-Old Serbian Children: A Comparison between 1990 and 2020" was published in 2022. Journal: Biomed Res Int.

In 1990, the average height (95% IP) of the 7-year-old boys was significantly lower in all morphological variables, compared to their 2020 peers, body height 2.6-5.3 cm and body mass 2.6-6.6 kg, as well as in BMI (*p* < 0.0001) and upper arm skinfold 5.2-7.5 cm, while in forearm circumference (1.1-10.3 cm) was opposite. As for the 11-year-old boys, body mass (*p* = 0.02) and BMI (0.009) had significantly better average values in 2020 than 1990, while in terms of forearm circumference (1.6-2.5 cm) and upper arm skinfold (2.7-4.9 cm), it was opposite. Differences in morphological characteristics between 7- and 11-year-old boys measured in 1990 and 2020 are presented in Table 2.

### 3.2. Morphological Characteristics of 7- and 11-Year-Old Girls (1990-2020)

In 1990, the average height (95% IP) of 7-year-old girls was between 126.5 and 127.8 cm, and body mass was from 26.17 to 17.19 kg, with BMI value of 16.55 ± 3.48 kg/m^2^. Their forearm circumference was between 17.36 and 17.66 cm, along with upper arm skinfold from 9.08 to 9.92 cm. Furthermore, the average height (95% IP) of 11-year-old girls was between 148.9 and 150.4 cm, and body mass was from 39.9 to 41.6 kg, with BMI value of 18.36 ± 4.38 kg/m^2^. Their forearm circumference was between 19.7 and 20.1 cm, along with upper arm skinfold from 10.9 to 11.8 cm. In 2020, 7-year-old girls' height (95% IP) was between 128.4 and 131.2 cm, and body mass varied from 27.73 to 31.73 kg, with BMI value of 17.86 ± 3.68 kg/m^2^. Their forearm circumference was between 19.56 and 36.78 cm, along with upper arm skinfold from 13.24 to 16.38 cm. Furthermore, 11-year-old girls' height (95% IP) was between 144.8 and 148.5 cm, and body mass was from 37.44 to 42.25 kg, with BMI value of 18.69 ± 4.78 kg/m^2^. Their forearm circumference was between 20.86 and 21.9 cm, along with upper arm skinfold from 11.56 to 16.74 cm.

Seven-year-old girls from a 1990 sample had significantly lower average values of morphological characteristics, compared to their 2020 peers: body height (*p* = 0.001), body mass (0.004), BMI (*p* = 0.009), forearm circumference (2-19.3 cm), and upper arm skinfold (3.7-7 cm). All morphological characteristic variables of 11-year-old girls have significantly better average values in 1990 than in 2020, except for body mass (*p* = 0.47) and BMI (*p* = 0.55). Body height in the 1990 sample was lower (1-5 cm), along with forearm circumference (1-2.1 cm) and upper arm skinfold (0.2-5.4 cm). Differences in morphological characteristics between 7- and 11-year-old girls measured in 1990 and 2020 are presented in Table 3.

The article "Trends in Morphological Characteristics among 7- and 11-Year-Old Serbian Children: A Comparison between 1990 and 2020" was published in 2022. Journal: Biomed Res Int.

### 3.3. Standardized Differences in Morphological Characteristics of 7- and 11-Year-Old Boys (1990-2020)

The average difference in body height (*g* = 0.7 [0.45, 0.94]) and body mass (*g* = 0.68 [0.34, 0.92]) of 7-year-old boys (1990-2020) is between large and small and in favor of 7-year-old boys from the year of 2020. As far as the BMI is concerned, the difference was small to moderate (*g* = −0.46 [-0.69, -0.24]). Likewise, the average difference between 7-year-old boys from 1990 and 2020 ranges from small to moderate in favor of the 2020 sample in forearm circumference (*g* = 0.52 [0.27, 0.76]). Seven-year-old boys from year of 2020 have presented much bigger average level of upper arm skinfold (*g* = 1.49 [1.23, 1.75]).

In 11-year-old boys, the differences in body height were trivial (*g* = 0.02 [-0.21, 0.24]) while in terms of body mass and BMI were trivial to moderate, respectively (*g* = 0.28 [0, 0.5]; *g* = −0.30 [-0.52, -0.08]). In addition, it was noted moderate to large differences in forearm circumference (*g* = 0.99 [0.75, 1.22]) as well as in upper arm skinfold (*g* = 0.76 [0.53, 0.98]). Hedge's *g* with 95% confidence interval for morphological differences between 7- and 11-year-old boys (1990-2020) are presented in Figure 1.

### 3.4. Standardized Differences in Morphological Characteristics of 7- and 11-Year-Old Girls (1990-2020)

The average differences in body height (*g* = −0.38 [-1.63, -0.12]) and BMI (*g* = −0.37 [-0.64, -0.11]) are trivial to moderate in a 1990 sample, respectively, while in the terms of body mass, the difference is only trivial (*g* = −0.09 [-0.35, 0.16]). Likewise, the average forearm circumference of 7-year-old girls is moderate than the 2020 sample (*g* = 0.75 [0.49, 1.01]), while the upper arm skinfold results are moderate than the 2020 sample (*g* = 0.36 [0.1, 0.62]).

In 11-year-old girls, the differences in body height (*g* = 0.47 [0.29, 0.65]), body mass (*g* = 0.5 [0.32, 0.68]), and forearm circumference (*g* = 0.53 [0.35, 0.71]) are between small and moderate than in the 2020 sample compared to the 1990 sample, while in terms of upper arm circumference, the 2020 sample is showing much higher values, compared to the 1990 sample (*g* = 1.08 [0.89, 1.26]). As far as the BMI is concerned, the difference was trivial (*g* = −0.07 [-0.33, 0.18]). Hedge's *g* with 95% confidence interval for morphological differences between 7- and 11-year-old girls (1990-2020) are presented in Figure 2.

## 4. Discussion

The study aim was to examine the current state, dynamics, and direction of changes in morphological characteristics, on a sample of 7- and 11-year-old Serbian children and adolescents, based on the first measurement that has been conducted 30 years ago. The main study findings are that average height (95% IP) of 7-year-old boys was significantly lower in all morphological variables in 1990, compared to their 2020 peers, while in forearm circumference was opposite. As for the 11-year-old boys, body mass (*p* = 0.02) and BMI (0.009) had significantly better average values in 2020 than 1990, whereas forearm circumference (1.6-2.5 cm) and upper arm skinfold (2.7-4.9 cm) results were opposite. Seven-year-old girls from a 1990 sample also had significantly lower average values of morphological characteristics, compared to their 2020 peers. All morphological characteristic variables of 11-year-old girls have significantly better average values in 1990 than 2020, except for body mass (*p* = 0.47).

The article "Trends in Morphological Characteristics among 7- and 11-Year-Old Serbian Children: A Comparison between 1990 and 2020" was published in 2022. Journal: Biomed Res Int.

The independent sample *t*-test revealed that significance in terms of 7-year-old boys and girls is shorter, lighter, and less adipose. Although boys showed a better trend in morphological characteristics, our study results agrees with the Kasović et al. [27], who also showed that boys have lower values of subcutaneous tissue mass and fat mass compared to girls. It should be noted that it is already a well-known fact that girls are more adipose than boys [28, 29]. In addition, it is necessary to take into account proper nutrition, adequate physical activity, sedentary activities, and sleep quality, since the negative impact on these parameters increases the possibility of overall health risk [30]. The result diversity can be also explained by the sample heterogeneity, age categories, statistical data processing, and even different time periods for estimating the secular trend of morphological parameters [31].

Significantly higher values of forearm circumference and skinfold were observed in favor of children from 2020, while body height and body mass did not differ significantly. Identical to 7 year olds, 11 year olds show an increased trend in morphological characteristics, and the results correspond to several studies as well [32–34]. On the other hand, between 1971 and 2018, Kocić et al. [35] determined a moderate effect of size in body height, for boys (*d* = 0.43) and for girls (*d* = 0.14), and in body mass, for boys (*d* = 0.5) and for girls (*d* = 0.62). However, due to the additional time point of measurement (2014), the same authors came to a significant effect size in the case of both genders. Meanwhile, between 1971 and 2014, the effect of body height was *d* = 1.28 for 11-year-old boys while for 11-year-old girls was *d* = 1.19. The case of body mass was *d* = 1.02 for 11-year-old boys while for 11-year-old girls was *d* = 1.04. Also, between 2014 and 2018, the effect of body height of both sexes was also large (boys: *d* = 0.85; girls: *d* = 1.19), as in the case of body mass (boys: *d* = 0.37; girls: *d* = 0.39). Božić-Krstić et al. [36] have also found an increased trend in body mass in 11-year-old children between 1971 and 1991, where the increased trend actually declined during 2001, most likely due to the economic situation at that period of time. Therefore, it is necessary to reconsider physical activities in physical education classes [37], both in Serbia and in other countries, based on the noticeable morphological changes. The fact that possible changes in school ergonomics could occure should also not be excluded [38], as well as a greater emphasis on more frequent and serious health status evaluations.

The article "Trends in Morphological Characteristics among 7- and 11-Year-Old Serbian Children: A Comparison between 1990 and 2020" was published in 2022. Journal: Biomed Res Int.

The results showed that all variables of morphological characteristics of 11-year-old boys had significantly better average values in 1990 than in 2020, except in the case of trivial differences in body height. In the case of 11-year-old girls in the 1990 sample, significant average values of all morphological characteristics were presented, except the body mass. Also, the results have showed increased body mass trend of children from 2020 (boys: *g* = 0.28; girls: *g* = 0.5). Since these differences are slightly more pronounced in boys than in girls, these results are consistent with Runhaar et al. [32]. In addition, based on the positive correlation and motor abilities with the maturity of boys and girls, we can say that maturity has an independent effect not only on physical fitness but also on the children's morphological structure [39]. Furthermore, there are fewer games that require any kind of movement, since today's children are spending more time at home sedentary, with some electronic devices (television, computer, or mobile phone) [40]. Therefore, if changes are not made in a certain period of time, difficulties can arise when the child completes the first grade [41], and when morphological difficulties occurs, there is a possibility that the negative trend will increase in the upper grades as well.

Based on the obtained results of the Hedge *g* test with 95% confidence interval for differences between morphological characteristics in relation to sex, children aged 7 years in 1990 and 2020, 7-year-old boys in 1990 show a positive trend in body height (*g* = 0.7), body mass (*g* = 0.68), upper arm skinfold (*g* = 1.49), and forearm circumference (*g* = 0.52). On the other hand, girls in 1990 were slightly taller (*g* = −0.38) and less adipose (forearm circumference: *g* = 0.75; upper arm skinfold: *g* = 0.36), with trivial differences in body mass (*g* = −0.09). Sedlak et al. [42] identified similar results on an identical sample over a period of 55 years. Namely, through 5 time point measurements, skinfolds (triceps, subscapular, and suprailiac) showed a significant positive trend in the case of both sexes, which partially agrees with our results. It should also be noted that the same study through two-time measurements (1957 and 1990) showed somewhat less significance; however, a more pronounced change in adiposity variables appeared during the last measurement (2012). Regarding body height and mass, development increased according to the time period of measurement [43], which also partially agrees with our results, since the body mass of girls changed trivially. If we take into account the time points of our study with Sedlak et al. [42], we should not ignore significant social and economic changes that have led to lifestyle changes, which further resulted in increased obesity prevalence [1].

The article "Trends in Morphological Characteristics among 7- and 11-Year-Old Serbian Children: A Comparison between 1990 and 2020" was published in 2022. Journal: Biomed Res Int.

Based on the obtained results of the Hedge *g* test with 95% confidence interval for differences between morphological characteristics in relation to sex, children aged 11 years in 1990 and 2020, boys have showed significantly better values of morphological characteristics, except in the case of body height (*g* = 0.02), while girls also showed significant average values of all morphological characteristics, except in the case of body mass (*g* = 0.5), in relation to the 2020 sample. The results presented in this way can be compared with the Costa et al. [33] results, who have presented significant differences over time in the variables of body mass but not in boys' body height. The same authors also identified significant changes in the body height and mass of girls, which partially agrees with our results. Differences in forearm circumference and upper arm skinfold agree with the results of Dollman and Stephen [44], and the same variables were more pronounced in girls than in boys. Variations in the results of morphological characteristics over time could be related to adequate diet and even eating habits, especially during the period when children are in school [45], which should be taken into consideration.

## 5. Conclusion

Reduced children's physical activity leads to a change in morphological characteristics. In addition, in certain stages of growth, the influence/interaction of genetic and environmental factors is not the same. The results of the current research have presented a true “picture” of the trends in morphological characteristics status among 7- and 11-year-old Serbian children by comparing them with the results from 30 years ago. From 1990 to 2020, we observed increase in height, body mass, and BMI in 7-year-old children. Although we have not included additional time points for morphological evaluation, as well as the fact that we have had included, only a few morphological variables could be considered as our main study limitations. Therefore, the conclusions regarding secular trends in morphological characteristics should include several time point measurements, along with more included morphological variables.

The article "Trends in Morphological Characteristics among 7- and 11-Year-Old Serbian Children: A Comparison between 1990 and 2020" was published in 2022. Journal: Biomed Res Int.

## Figures and Tables

**Figure 1:** Standardized differences in morphological characteristics of 7- and 11-year-old boys. Legend: BH: body height; BM: body mass; BMI: body mass index; FC: forearm circumference; UAS: upper arm skinfold.

**Figure 2:** Standardized differences in morphological characteristics of 7- and 11-year-old girls. Legend: BH: body height; BM: body mass; BMI: body mass index; FC: forearm circumference; UAS: upper arm skinfold.

**Table 1:** The number of participants in both time points.

Year	Participant sample	
1990	*n*_7_ = 858 (M = 430; F=428)	∑ = 1789
	*n*_11_ = 931 (M = 455; F = 476)	

2020	*n*_7_ = 143 (M = 79; F = 64)	∑ = 304
	*n*_11_ = 161 (M = 94; F = 67)	

Legend: *n*_7_: 7-year-old participants; *n*_11_: 11-year-old participants; M: male; F: female; ∑: total number of participants.

**Table 2:** Morphological characteristics in 7- and 11-year-old boys measured 1990 and 2020.

Variables	Age	Mean ± SD		*p*
		1990	2020	
BH (cm)	7	127.78 ± 5.94	131.73 ± 5.37	<0.001
	11	147.55 ± 7.53	147.67 ± 7.45	0.888

BM (kg)	7	27.28 ± 4.86	31.89 ± 8.76	<0.001
	11	40.35 ± 9.23	43.06 ± 10.30	0.020

BMI (kg/m^2^)	7	16.91 ± 3.63	18.58 ± 3.57	<0.001
	11	18.67 ± 4.11	19.93 ± 4.71	0.0096

FC (cm)	7	17.73 ± 1.53	23.43 ± 20.48	0.016
	11	20.23 ± 1.97	22.27 ± 2.13	<0.001

UAS (cm)	7	8.54 ± 3.57	14.89 ± 4.95	<0.001
	11	10.78 ± 5.40	14.58 ± 4.63	<0.001

Legend: BH: body height; BM: body mass; BMI: body mass index; FC: forearm circumference; UAS: upper arm skinfold; SD: standard deviation; *p*: *p* value.

**Table 3:** Morphological characteristics in 7- and 11-year-old girls measured 1990 and 2020.

Variables	Age	Mean ± SD		*p*
		1990	2020	
BH (cm)	7	127.15 ± 6.4	129.75 ± 5.62	<0.001
	11	149.63 ± 8.24	146.65 ± 7.56	0.004

BM (kg)	7	26.68 ± 5.36	29.73 ± 7.99	0.004
	11	40.76 ± 9.42	39.84 ± 9.86	0.474

BMI (kg/m^2^)	7	16.54 ± 3.48	17.86 ± 3.68	<0.001
	11	18.36 ± 4.38	18.69 ± 4.78	0.55

FC (cm)	7	17.51 ± 1.53	28.17 ± 34.47	0.016
	11	19.85 ± 1.95	21.38 ± 2.12	<0.001

UAS (cm)	7	9.45 ± 3.94	14.81 ± 6.28	<0.001
	11	11.36 ± 4.85	14.15 ± 10.62	0.038

Legend: BH: body height; BM: body mass; BMI: body mass index; FC: forearm circumference; UAS: upper arm skinfold; SD: standard deviation; *p*: *p* value.

The article "Trends in Morphological Characteristics among 7- and 11-Year-Old Serbian Children: A Comparison between 1990 and 2020" was published in 2022. Journal: Biomed Res Int.

## Data Availability

The data presented in this study are available on request from the corresponding author.
